# Long Noncoding RNA LINC01503 Silencing Suppresses KLK4 Expression to Impede Pancreatic Cancer Development as miR-1321 Sponge

**DOI:** 10.1155/2023/5403344

**Published:** 2023-02-04

**Authors:** Baiping An, Yi Cai, Jie Zhu, Yuan Liu

**Affiliations:** ^1^Department of Oncology, Hospital of Chengdu University of Traditional Chinese Medicine, Chengdu City 610032, China; ^2^Department of Interventional Oncology, Hospital of Chengdu University of Traditional Chinese Medicine, Chengdu City 610032, China

## Abstract

**Background:**

Long intergenic nonprotein coding RNA 1503 (LINC01503) was reportedly oncogenic in several malignancies, whereas whether it contributed to pancreatic cancer tumorigenesis and progression requires to be verified.

**Methods:**

The expression pattern of LINC01503 was monitored via qRT-PCR assay in normal cells and cancerous pancreatic cancer cells. The introduction of silencing LINC01503 was to verify the relation between LINC01503 expression and cell growth. Then, the targeting relationship of LINC01503 to miR-1321 was confirmed by bioinformatics predication and luciferase reporter assay. In addition, luciferase reporter assays evaluated the binding of miR-1321 to the 3′-untranslated region of KLK4. Overexpressing KLK4 and inhibiting LINC01503 was introduced in tumor cells to investigate the corresponding impacts on pancreatic cancer cell proliferation and migration.

**Results:**

LINC01503 and KLK4 were highly abundant in pancreatic cancer cells. Mechanistically, miR-1321 bound to LINC01503 and KLK4. Downregulating LINC01503 promoted the availability of miR-1321 in pancreatic cancer cells and thus repressed KLK4 expression. KLK4 overexpression abolished the impediment of LINC01503 depletion on cell proliferation and migration.

**Conclusion:**

Oncogenic function of LINC01503 was dependent on KLK4 upregulation by sponging miR-1321. Revealing the tumor-promoting property of LINC01503 in pancreatic cancer may confer new biomarkers for this malignancy.

## 1. Introduction

Pancreatic cancer (PC) has attracted widespread attention since it accounted for the most cancer-related mortality and the consequent cancer invasion and aggressiveness [1, 2]. One outstanding feature of PC is the desmoplastic/stromal reaction, and it was ultimately recognized as a fatal malignancy by the discouraging 5-year survival rate [3, 4]. Due to the lack of screening image modalities and efficient biomarkers, inefficient early diagnosis brings about the stumbling block for PC control [5]. Furthermore, the unfavorable outcomes frequently occur owing to adverse factors such as metastasis and drug resistance. Accordingly, developing more innovative and feasible treatment strategies is in urgent necessity for PC [5].

Long noncoding RNAs (lncRNAs) are sized 200 nt and recently identified as noncoding RNAs with restricted open reading frame [6]. Initially, scare attention was paid to lncRNAs, but gradually increasing research has focused on the essential functions of lncRNAs in the cell growth, apoptosis, cell cycle, differentiation, and eventually disease pathogenesis [7, 8]. lncRNAs have been uncovered to be abnormally expressed during the cellular processes of cancer development. For instance, lncRNA GNAT1-1 is expressed at a low level in colorectal cancer and behaves as a tumor inhibitor [9]. The overexpressed lncRNA MIR155HG contributes to the cell growth and progression of glioblastoma [10]. lncRNA FEZF1-AS1 is highly expressed and accelerates proliferation and metastasis in colorectal tumor through regulating PKM2 signaling [11]. Mechanistically, the binding ability of lncRNAs to specific microRNAs (miRNAs) was widely certified to contribute to target gene expression [12]. For example, lncRNA GAPLINC is capable of sponging miR211-3p from CD44 to facilitate cell invasiveness and predicts poor prognosis of gastric cancer [13]. lncRNA DANCR acts as a bladder cancer facilitator through sponging miR-149and upregulating MSI2 expression [14]. lncRNA MIR31HG serves as a hepatocellular carcinoma inhibitor by acting as a microRNA-575 sponge and modulating ST7L expression [15].

It has been implied in previous literature that long intergenic nonprotein coding RNA 1503 (LINC01503) is a tumor driver [16–18]. It has also been unveiled as a significantly upregulated lncRNA in PC from TCGA dataset on GEPIA website (http://gepia2.cancer-pku.cn/#index). However, valuable information about its function or mechanism in PC has been inadequate so far. The present study tried to investigate its expression pattern in PC cells. After the construction of LINC01503 knockdown plasmids, we explored the influence of LINC01503 downregulation on PC cell proliferation, migration, and epithelial mesenchymal transition (EMT). Through bioinformatics prediction and mechanistic assays, the regulatory mechanism of LINC01503 was also delved. We attempted to figure out if LINC01503 acted as a competing endogenous RNA (ceRNA) to mediate downstream target-dependent cell growth and mobility through sponging a certain miRNA. Altogether, our study elucidated the pivotal function of LINC01503 and meanwhile depicted the regulatory axis of LINC01503 in PC cells, offering a new direction in developing promising therapeutic targets for PC patients.

## 2. Materials and Methods

### 2.1. Cell Lines and Culture

PC cells (PANC-1, AsPC-1, SW1990, and BxPC-3) and noncancerous pancreatic cells (HPDE6-C7) were obtained from American Type Culture Collection (ATCC, USA). Cell lines used in this study were cultured in Dulbecco's modified Eagle's medium (DMEM, Gibco) with 10% FBS maintained in a humidified incubator at 37°C containing 5% CO_2_ according to the specifications.

### 2.2. Cell Transfection

AsPC-1 and SW1990 with higher expression of LINC01503 than the other PC cells were selected to conduct the transfection. Short hairpin RNAs (shRNAs) targeting LINC01503 (sh-LINC01503#1/2) with the corresponding negative control (sh-NC), miR-1321 mimics/inhibitors, their matched controls (NC-mimics/NC-inhibitor), LINC01503-overexpressing plasmids (pcDNA3.1/LINC01503), and KLK4-overexpressing plasmids (pcDNA3.1/KLK4), along with the empty plasmids (pcDNA3.1), were all supplied by RiboBio Co. (Guangzhou, China). Transfection of AsPC-1 and SW1990 cells with indicated plasmids was conducted referring to the manufacturer's protocols of Lipofectamine® 2000 (Invitrogen; Thermo Fisher Scientific, Inc.).

### 2.3. RNA Extraction and Quantitative Real-Time Polymerase Chain Reaction (qRT-PCR) Assay

RNA extraction was carried out in cell samples following the supplier's instructions of TRIzol reagent (Invitrogen; Thermo Fisher Scientific, Inc.). To measure RNA expression, complementary DNA (cDNA) was synthesized utilizing Roche Transcriptor First Strand cDNA Synthesis kit (Hengfei, Minhang, Shanghai, China). Subsequently, on a QuantStudio 12 K Flex Real-Time PCR apparatus (ORST, Chengdu, China), the qRT-PCR assay was implemented applying a SYBR Green qPCR Master Mix (MedChemExpress, Pudong, Shanghai, China). The method of 2^-*ΔΔ*Ct^ was applied for the quantification of RNA expression. GAPDH was used for normalization as endogenous controls of lncRNA and mRNA and U6 for miRNAs. The primer sequences used in this research are listed in Table 1.

### 2.4. Cell Counting Kit-8 (CCK-8) Assay

The 96-well plates (l00 *μ*L/well) were seeded with PC cells (AsPC-1 and SW1990) at the density of 1 × l0^4^ cells/well, and cells underwent transfection. Subsequently, l0 *μ*L CCK-8 solution was supplemented in each well at the 24th, 48th, and 72th hour. Afterward, PC cells were preserved in a cell incubator for 4 hours. A microplate reader set at 450 was used for reading the absorbance value.

### 2.5. 5-Ethynyl-20-Deoxyuridine (EdU) Assay

The proliferation capacity of AsPC-1 and SW1990 cells was evaluated through this assay. The abovementioned PC cells were first planted into 48-well plates and transfected with indicated plasmids. Forty-eight hours later, a Cell-Light Cell Proliferation kit (RiboBio, Guangzhou, Guangdong, China) was utilized, followed by the incubation with EdU reagent (50 *μ*M) for 2-3 hours. Subsequently, the cell nuclei were stained for 10 minutes with DAPI (1 *μ*g/mL). Finally, an inverted fluorescence microscope (HGO, Suzhou, Jiangsu, China) was applied for observing fluorescence signals of those cells after treatments.

### 2.6. Terminal Deoxynucleotidyl Transferase Mediated Nick End Labeling (TUNEL) Assay

An in situ Cell Death Detection Kit (ROCHE, USA) required for TUNEL assay was applied to investigate AsPC-1 and SW1990 cell apoptosis in this study. The 1% polytetrafluoroethylene was utilized for fixing the cell samples at room temperature in phosphate-buffered saline (PBS; HyClone) for 10minutes, and the immobilized cells later underwent cooled ethanol permeabilization, followed by immersing cells in equilibration buffer. Next, cells after working strength TdT enzyme treatment were incubated for an hour at 37°C. Then, the reaction was stopped through the addition of top buffer. The cells cleaned by PBS were incubated in the dark with antidigoxigenin conjugate for 30 minutes at room temperature.

### 2.7. Transwell Assay

To probe AsPC-1 and SW1990 cell migration, the upper chamber was cultured in the cell incubator for 4 hours. After the preparation of the cell suspension, it was seeded into the apical chamber. The bottom chamber was filled with 0.5 mL DMEM containing 10% FBS as the chemotactic inducer. Following the 8 h incubation, nonpenetrating cells were wiped off gently by swab, followed by a 15 min of fixation and 0.1% crystal violet staining. The cells that migrated to the bottom compartment were counted with a high-magnification inverted microscope from 5 randomly selected fields.

### 2.8. Wound Healing Assay

PC cell samples following transfection were well maintained under appropriate conditions. In this assay, creation of the wounds was achieved by the means of a plastic scriber for the scratch of the cell monolayer. Subsequently, DMEM containing 10% FBS was employed for the 24 h incubation of AsPC-1 and SW1990 cells. A microscope was required for recording the migration activity of cells at 0 h and at 24 h. Determination of cell migration activity is conducted via the subtraction of the final wound width from the width at the beginning.

### 2.9. Western Blot Assay

The logarithmically growing AsPC-1 and SW1990 cells were firstly rinsed twice by ice-cold PBS, and then, radio-immunoprecipitation assay (RIPA) solution was applied for protein extraction. Under denaturing conditions, 10% sodium dodecyl sulphate-polyacrylamide gel electrophoresis (SDS-PAGE) was adopted for total protein separation and transferred to nitrocellulose membranes. The 5% skimmed milk was utilized for blocking the membranes, and later at 4°C, overnight membrane incubation with primary antibodies was conducted. Primary antibodies are anti-KLK4 (Abcam), anti-N-cadherin (Abcam), anti-vimentin (Abcam), and anti-GAPDH (Abcam). Tris-buffered saline and Tween (TBST) washed these membranes 3 times, and the washed membranes were incubated at room temperature with defined secondary antibody for an hour. Enhanced chemiluminescence (ECL) system was for exposing the immunoreactive bands.

### 2.10. Luciferase Reporter Assay

The binding affinity between miR-1321 and LINC01503/KLK4 on the basis of bioinformatics prediction was corroborated by this assay. Wild types of LINC01503 and KLK4 containing miR-1321 binding sites were first amplified and then cloned into psi-CHECKTM-2 vector (Promega, Madison, WI) for the construction of LINC01503-WT and KLK4-WT reporters. Then binding sites of miR-1321 in KLK4 and LINC01503 were mutated through the application of a GeneArt™ Site-Directed Mutagenesis PLUS System (Thermo Fisher Scientific, Inc.) to establish LINC01503-MUT and KLK4-MUT reporters by inserting LINC01503 and KLK4 sequence containing mutated miR-1321 binding sites into the psi-CHECKTM-2 vector. The indicated reporters and miR-1321 mimics/NC-mimics were cotransfected into AsPC-1 and SW1990 cells and incubated for 48 h to examine the combination of miR-1321 and LINC01503/KLK4. The pcDNA3.1/LINC01503 or pcDNA3.1 plasmids were cotransfected with KLK4-WT and miR-1321 mimics/NC-mimics to explore if LINC01503 competed with KLK4 to bind with miR-1321. Dual-Luciferase Reporter Assay System (Promega Corp.) was subsequently used for measuring the luciferase activities. The internal reference was the activity of Renilla.

### 2.11. RNA Immunoprecipitation (RIP) Assay

By means of a Magna RIP RNA-Binding Protein IP Kit (Millipore), this assay was accomplished on the basis of the manufacturer's specifications. Cell samples were lysed utilizing RIP lysis buffer. Subsequently, the cell lysates were incubated with specific primary antibody (anti-Ago2 and anti-IgG as NC) attained from Abcam. Magnetic beads were added for the incubation at 4°C overnight. Following purification, the detection of qRT-PCR was sequentially designed for the analysis of the coprecipitated RNAs.

### 2.12. Subcellular Fractionation Assay

The separation of cytoplasmic and nuclear fractions of AsPC-1 and SW1990 cells was completed with the use of a PARIS kit (Life Technologies) to investigate the subcellular location of LINC01503 in PC cells. The extracted RNA subsequently underwent the detection of qRT-PCR.U6 and GAPDH that were utilized as nuclear control and cytoplasmic control, respectively.

### 2.13. Statistical Analysis

The SPSS 21.0 software (IBM Corp. Armonk, NY, USA) was employed for statistics processing, and the quantitative data were demonstrated in the form of mean ± standard deviation (SD). Methods of Student's *t*-test and one-way/two-way analysis of variance (ANOVA) were applied for data comparison. In this regard, differences between two groups were analyzed by Student's *t*-test while difference analysis of multiple groups with one or two variables required ANOVA. When the *p* value was less than 0.05, the data differences represented to be statistically significant.

## 3. Results

### 3.1. LINC01503 Was Cytoplasmically Located and Overexpressed in PC Cells

For the functional identification of LINC01503 in pancreatic cancer, we searched LINC01503 expression patterns in pancreatic adenocarcinoma (PAAD) tissues and the adjacent normal tissues from GEPIA database. As presented in Figure 1(a), LINC01503 displayed a high expression in PAAD tumor tissues. Herein, we also found that in comparison of human pancreatic duct epithelial cells (HPDE6-C7), LINC01503 was upregulated in PC cells (AsPC-1, BxPC-3, SW1990, and PANC-1), especially in AsPC-1 and SW1990 cells (Figure 1(b)). The distribution of lncRNAs is closely associated with prognosis of PC and specific molecular mechanism [19]. Accordingly, through lncLocator (http://www.csbio.sjtu.edu.cn/bioinf/lncLocator/), it was projected that LINC01503 was primarily localized in the cytosol (Figure 1(c)). Consistently, subcellular fractionation assay also unveiled that LINC01503 was largely accumulated in PC cell cytoplasm (Figure 1(d)). To sum up, LINC01503 displayed a high expression in PC cells and primarily accumulated in the cell cytoplasm.

### 3.2. LINC01503 Silencing Suppressed PC Cell Growth and Facilitated Apoptosis

Prior to investigating the biological function of LINC01503 in PC cells, sh-LINC01503 plasmids were first confirmed to successfully downregulate LINC01503 (Figure 2(a)). Subsequently, CCK-8 and EdU assays uncovered that PC cell viability and proliferation were hampered due to LINC01503 depletion (Figures 2(b) and 2(c)). On the contrary, the proportion of apoptotic cells was higher in LINC01503-depleted PC cells compared with control group (Figure 2(d)). Collectively, LINC01503 depletion resulted in the suppression of PC cell proliferation and acceleration of the cell apoptosis.

### 3.3. LINC01503 Knockdown Led to Repressed PC Cell Migration

As a pivotal aspect of tumor progression, PC cell migration was also assessed in the absence of LINC01503. Through Transwell and wound healing assays, we observed that LINC01503 deficiency accounted for the inhibition of PC cell migration (Figures 3(a) and 3(b)). EMT is also a facilitator for the metastasis of tumor cells originated from epithelial cells [20, 21]. Subsequently, we detected the EMT-related protein levels in PC cells upon LINC01503 downregulation. Western blots manifested that LINC01503 knockdown led to a decrease of vimentin and N-cadherin protein contents (Figure 3(c)), which represented the impeded PC cell migration in response to LINC01503 inhibition.

### 3.4. LINC01503 Competed with KLK4 to Bind with miR-1321

Increasing evidence has suggested that cytoplasmic lncRNAs can function as a ceRNA to sponge miRNAs and indirectly upregulate downstream mRNAs [22]. Accordingly, we applied DIANA (http://carolina.imis.athena-innovation.gr/diana_tools/web/index.php?r=site%2Ftools) and starBase (http://starbase.sysu.edu.cn/) to predict the potential miRNAs probably binding with LINC01503. Venn diagram exhibited three putative miRNAs (miR-4756-5p, miR-1321, and miR-4739) as potential targets of LINC01503 (Figure 4(a)). Furthermore, we noticed that only miR-1321 was increased in response to LINC01503 depletion, while no obvious changes were observed in miR-4756-5p and miR-4739 expressions (Figure 4(b)). In addition, luciferase reporter assay corroborated the combination and binding sites between LINC01503 and miR-1321, as the luciferase activity of LINC01503-WT was reduced, rather than that of LINC01503-MUT (Figure 4(c)). Moreover, RIP assay reflected that LINC01503 and miR-1321 could be detected in anti-Ago2, evidencing the coexistence of LINC01503 and miR-1321 in the RNA-induced silencing complex (RISC) (Figure 4(d)). Through the bioinformatics analysis of TargetScan (http://www.targetscan.org/vert_72/) and miRDB (http://mirdb.org/), KLK4 stood out to be the downstream target highly associated with miR-1321, and the predicted binding sites are shown (Figure 4(e)). Western blots demonstrated that KLK4 protein level was significantly upregulated in PC cells, relative to HPDE6-C7 cells (Figure 4(f)). It was also observed that miR-1321 elevation suppressed the luciferase activity of KLK4-WT but did not impact that of KLK4-MUT (Figure 4(g)). In addition, the high efficacy of LINC01503 overexpression plasmids was synthesized and determined to be efficient (Figure S1A). Luciferase reporter assay further uncovered that LINC01503 augmentation could restore the reduced luciferase activity of KLK4 caused by miR-1321 upregulation. This finding indicated that LINC01503 competed with KLK4 to sequester miR-1321 (Figure S1B). Moreover, we found that miR-1321 negatively regulated KLK4 expression (Figure 4(h)). Noteworthily, the inhibitory impact of LINC01503 deficiency on KLK4 mRNA and protein levels was abrogated by miR-1321 inhibition (Figures 4(i) and 4(j)). The abovementioned data elaborated that LINC01503 competitively bound with miR-1321 and positively modulated KLK4 expression.

### 3.5. LINC01503 Regulated PC Cell Growth and Migration via KLK4

In this part, we tried to explore the regulation of LINC01503/KLK4 axis on PC cell growth and migration. Augmentation of KLK4 in PC cells was validated (Figure 5(a)). CCK-8 and EdU assays uncovered that KLK4 overexpression abrogated the suppressive influence of LINC01503 downregulation on PC cell viability and proliferation (Figures 5(b) and 5(c)). The diminished number of migrated PC cells was caused by LINC01503 reduction that was also recovered after pcDNA3.1/KLK4 transfection (Figure 5(d)). Consistently, the inhibited PC cell migration resulting from LINC01503 deficiency was restored by KLK4 overexpression (Figure 5(e)). Western blot assay further presented that the levels of EMT-associated proteins decreased by LINC01503 knockdown which rose again on account of KLK4 increment (Figure 5(f)). The aforementioned findings suggested that LINC01503 modulated PC cell growth and migration through upregulating KLK4.

## 4. Discussion

For decades, the dysregulation of numerous lncRNAs was elaborated to be responsible for the carcinogenesis and aggravation of multiple malignancies with the advances made in cancer research [23]. Lately, LINC01503 has been unveiled as an oncogenic inducer in squamous cell carcinoma on account of TP63 upregulation [17]. LINC01503 has also been proven as a promoter for colorectal cancer cell proliferation and invasion through the elevation of FOXK1 and the inhibition of miR-4492 [16]. According to another research work, LINC01503 is able to activate Wnt/*β*-catenin signaling to facilitate glioma tumorigenesis as well as progression and predict adverse clinical outcomes [18]. Previous literature evidences that LINC01503 is tumor promoting in diverse tumors. Through the exploration in TCGA datasets, we also found LINC01503 was upregulated in PC tissues compared with normal tissue samples. In our study, the elevated level of LINC01503 in PC cell was also observed. Functional assays illuminated that LINC01503 knockdown resulted in inhibited PC cell viability, proliferation, migration, and EMT process, which was consistent with the proproliferation and migration function documented previously but was first corroborated in PC development.

Mechanistically, the posttranscriptional modulation of lncRNA as a ceRNA has also received extensive investigation that lncRNAs sponged miRNAs and decreased its inhibitory activity for target genes [24]. This regulatory mediation of lncRNAs in fact has also been introduced in PC. For instance, LINC00511 enhances VEGFA expression through the ceRNA function on miR-29b-3p to aggravate PC development [25]. lncRNA SNHG16 contributes to PC tumor growth by targeting miR-218-5p and further boosting HMGB1 expression [26]. lncRNA AFAP1-AS1 promotes PC cell growth and invasion through overexpressing IGF1R oncogene via sequestering miR-133a [27]. It has also been verified that LINC01503 acts as a sponge for miR-4492 to upregulate FOXK1 expression [16]. In this research, we focused on identifying the role of LINC01503 as a ceRNA. Through bioinformatics analysis and mechanistic experiments, miR-1321 was proved to interact with and suppressed by LINC01503; the targeting relationship between LINC01503 and miR-1321 was first substantiated in PC.

On the other hand, targets of miR-1321 were also determined through online prediction and experimental validation. We identified KLK4 as the candidate target of miR-1321. Published work has well explained that KLK4 is conducive to malignant tumor phenotype, such as proliferation and migration in various cancers. For example, KLK4 boosts oral squamous cell carcinoma metastasis and progression [28, 29]. KLK4 has also been proven to be proliferative in prostate cancer [30]. Currently, documentation about its involvement or function in PC was limited. Consistent with our hypothesis, KLK4 was found to be abundant in PC cells and competed with LINC01503 to bind with miR-1321. The implied oncogenic role of KLK4 was further exemplified in the later rescue experiments, in which KLK4 augmentation was capable of abrogating the suppressive trend of cell proliferation and migration caused by LINC01503 depletion.

In summary, it was clarified that LINC01503 was highly expressed in PC cells, and its silencing led to the inhibition of cell growth and migration. Most importantly, it was the first documentation that LINC01503 depended on KLK4 elevation via sponging miR-1321 to facilitate PC progression. Although clinical samples and in vivo study were not involved in this study, our findings might provide a novel strategy of targeting LINC01503 in early diagnosis of PC.

## Figures and Tables

**Figure 1:** LINC01503 was cytoplasmically located and overexpressed in PC cells. (a) GEPIA database presented the expression pattern of LINC01503 in PC tissues and normal tissues. (b) LINC01503 expression in PC cells and normal pancreatic cells were examined through qRT-PCR. (c) lncLocator website predicted the location of LINC01503 in cells. (d) Subcellular fractionation assay detected LINC01503 distribution in PC cells. ^∗^*p* < 0.05.

**Figure 2:** LINC01503 silencing suppressed PC cell growth and promoted apoptosis. (a) The efficacy of LINC01503 knockdown was tested through qRT-PCR. (b) PC cell viability was analyzed by CCK-8 assay after silencing LINC01503. (c) EdU assay detected the impact of LINC01503 knockdown on PC cell proliferation. (d) TUNEL assay monitored PC cell apoptosis after LINC01503 inhibition. ^∗^*p* < 0.05, ^∗∗^*p* < 0.01, and ^∗∗∗^*p* < 0.001.

**Figure 3:** LINC01503 knockdown led to the inhibition of PC cell migration. (a, b) Transwell and wound healing assay investigated PC cell migration upon LINC01503 silencing. (c) Western blot assay measured vimentin and N-cadherin proteins in LINC01503-depleted PC cells. ^∗∗^*p* < 0.01.

**Figure 4:** LINC01503 competed with KLK4 to sequester miR-1321. (a) Three candidate miRNAs possibly interacting with LINC01503 were predicted by DIANA and starBase databases. (b) qRT-PCR examined the expression of candidate miRNAs upon LINC01503 knockdown. (c) The binding sites of LINC01503 on miR-1321 were shown, and luciferase reporter assay evaluated the combination of LINC01503 and miR-1321. (d) RIP assay detected the enrichment of LINC01503 and miR-1321 in anti-Ago2. (e) The TargetScan and miRDB databases predicted the binding affinity and binding sequence of miR-1321 to KLK4. (f) Western blot examined KLK4 protein level in PC cells and normal pancreatic cells. (g) Luciferase reporter assay examined the combination of miR-1321 and KLK4. (h) Effects of miR-1321 upregulation or inhibition on KLK4 expression were detected through qRT-PCR. (i, j) qRT-PCR and western blot assays monitored KLK4 mRNA and protein levels in PC cells upon indicated transfections. ^∗^*p* < 0.05, ^∗∗^*p* < 0.01, and ^∗∗∗^*p* < 0.001.

**Figure 5:** LINC01503 regulated PC cell growth and migration via KLK4. (a) KLK4 overexpression efficiency was confirmed by qRT-PCR assay. PC cells were grouped according to indicated plasmids, including sh-NC, sh-LINC01503#1, sh-LINC01503#1+pcDNA3.1, and sh-LINC01503#1+pcDNA3.1/KLK4. (b, c) CCK-8 and EdU assays measured PC cell viability and proliferation under different conditions. (d, e) Migratory ability of PC cells was estimated by Transwell and wound healing assays. (f) Western blot assay detected EMT-related protein levels in PC cells after indicated transfections. ^∗^*p* < 0.05 and ^∗∗^*p* < 0.01.

**Table 1:** Primer sequences used in this study.

Gene name	Sequence (F: forward primer; R: reverse primer)
LINC01503	F: GTGATGCTGATGTGTGACTGC
	R: ACCTAGGGCTCTGCATTCGT

miR-4756-5p	F: CCGAGcagggaggcgctcactc
	R: CTCAACTGGTGTCGTGGA

miR-4739	F: CCGAGaagggaggaggagcggagg
	R: CTCAACTGGTGTCGTGGA

miR-1321	F: CCGAGcagggaggtgaa
	R: CTCAACTGGTGTCGTGGA

KLK4	F: CGCACACTGTTTCCAGAACTC
	R: GTTAGCGAGCAAGGGTCTGT

GAPDH	F: GTCAAGGCTGAGAACGGGAA
	R: AAATGAGCCCCAGCCTTCTC

U6	F: TCCCTTCGGGGACATCCG
	R: AATTTTGGACCATTTCTCGATTTGT

## Data Availability

The data used to support the findings of this study are included within the article.

## Supplementary Materials

Supplementary Materials Figure S1: (A) the efficacy of LINC01503 augmentation was tested through qRT-PCR. (B) Luciferase reporter assay assessed the competitive binding relationship among LINC01503, miR-1321, and KLK4 in PC cells. ^∗∗^*p* < 0.01.
